The article "A Multifeature Extraction Method Using Deep Residual Network for MR Image Denoising" was published in 2020. Journal: Comput Math Methods Med.

# A Multifeature Extraction Method Using Deep Residual Network for MR Image Denoising

**DOI:** 10.1155/2020/8823861

**Published:** 2020-11-05

**Authors:** Li Yao

**Affiliations:** School of Computing, Hubei Polytechnic University, Huangshi, Hubei 435003, China

## Abstract

In order to improve the resolution of magnetic resonance (MR) image and reduce the interference of noise, a multifeature extraction denoising algorithm based on a deep residual network is proposed. First, the feature extraction layer is constructed by combining three different sizes of convolution kernels, which are used to obtain multiple shallow features for fusion and increase the network's multiscale perception ability. Then, it combines batch normalization and residual learning technology to accelerate and optimize the deep network, while solving the problem of internal covariate transfer in deep learning. Finally, the joint loss function is defined by combining the perceptual loss and the traditional mean square error loss. When the network is trained, it can not only be compared at the pixel level but also be learned at a higher level of semantic features to generate a clearer target image. Based on the MATLAB simulation platform, the TCGA-GBM and CH-GBM datasets are used to experimentally demonstrate the proposed algorithm. The results show that when the image size is set to 190 × 215 and the optimization algorithm is Adam, the performance of the proposed algorithm is the best, and its denoising effect is significantly better than other comparison algorithms. Especially under high-intensity noise levels, the denoising advantage is more prominent.

## 1. Introduction

With the rapid development of information technology and computer vision, different digital imaging technologies emerge endlessly. An image has become one of the most common information transmission carriers in modern life. Up to now, the research on medical imaging has made some progress and achievements [1]. For example, methods such as positron emission tomography (PET), computer tomography (CT), magnetic resonance imaging (MRI), and functional magnetic resonance imaging (FMRI) have been used. They have become the main technical means for obtaining medical images. They have been successfully applied in clinical medical diagnosis [2]. These imaging technologies can enrich the anatomical images of clinical symptoms and can observe various lesions of the human body more clearly. It is conducive to image postprocessing and provides an important reference for clinical development. Image digital imaging technology is based on computers; collects, displays, stores, and transmits images to digitize image information; and optimizes each part individually. Electronic information, computer technology [3], and digital image processing methods are the basis of the above imaging technology. Using imaging technology to effectively complement the image information can achieve the effect of easy access to medical image information. It is helpful for clinicians to formulate treatment plans through image diagnosis acquisition, so as to accelerate the rapid development of medical research and new medical technology [4].

Among many medical imaging technologies, MRI is a high-resolution medical imaging technology for human tissues and organs. It can image various parts of the human body at multiple angles and in all directions and can obtain relatively complete medical image information [5]. For a complete image information processing system, it mainly includes modules such as information acquisition, information processing, information transmission, and information reception. However, in each of these links, the image may be polluted by the random noise of the Rician distribution. These noises reduce the signal-to-noise ratio of the image, which makes it difficult for doctors to distinguish the details of the lesion from the background [6]. In addition, noisy images will not only affect the visual effect but also adversely affect subsequent image analysis, such as image segmentation, target recognition, and edge detection. Therefore, it is very necessary to remove the noise in an image. Due to the lack of relevant research in the field of denoising, the postprocessing of an image is seriously affected, and the accuracy and effectiveness of imaging are reduced. Therefore, image denoising processing is particularly important [7].

An image denoising algorithm can effectively filter out image noise and at the same time enhance the useful information of the image [8]. That is, while eliminating image noise, the details of the image are preserved as much as possible. Image detail information is selectively strengthened and suppressed, and the edge of the image is highlighted, thereby improving the visual effect of the image [9]. When traditional image denoising methods filter medical MR image noise, it is easy to lose the edge information of the image and it is difficult to save the detailed information of the image, which is far from meeting the needs of medical diagnosis [10]. Therefore, there is an urgent need for new research methods and means to solve this problem.

## 2. Related Research

Image denoising is a difficult problem in the field of image processing. In order to get a clear image and effectively remove the noise introduced in the process of image generation, many domestic and foreign researchers have done a lot of research and put forward many very clever denoising algorithms. Some of the traditional image denoising methods have been proposed for a long time and have been widely used. However, most algorithms will inevitably damage the original useful information while denoising. And many algorithms need to be improved in denoising performance and model complexity [11]. How to strip out the noise and achieve a good denoising effect even under high-intensity noise has brought new challenges to the research of existing denoising algorithms. For medical MRI denoising algorithms, the more common ones are traditional image denoising algorithms, dual-domain filtering image denoising algorithms, and deep learning image denoising algorithms [12].

According to the denoising of traditional image denoising algorithms in different domains, these methods are divided into spatial domain and transform domain image denoising algorithms. In the image denoising algorithm in the spatial domain, the commonly used spatial domain filtering methods mainly include mean filtering, median filtering, and Wiener filtering [13]. The mean filter is a linear smoothing filter, which can effectively deal with the additive white Gaussian noise in the image. In Reference [14], an effective image denoising method is proposed for images damaged by salt and pepper noise. A modified mean filter (MMF) is used to restore the image by processing the value. For serious noise damage, the noise pixel value is replaced by the weighted average value of MMF sum. The change of damaged pixels can be minimized by convex optimization, and two fuzzy systems are used to determine the weight of the average value to achieve denoising. The mean filter is equivalent to a low-pass filter. Although the operation is simple and the calculation speed is fast, the mean filter will lose the details in the denoising process and make the image blurry [15]. Median filtering was originally a nonlinear processing technique used to analyze time series and was later used to remove salt and pepper noise. Wiener filtering can better filter out salt and pepper noise through the local statistical characteristics of the image according to the minimum mean square error. In Reference [16], an improved Wiener filtering method is proposed to denoise satellite images. Different noise and filtering techniques are studied in detail, and the results show that the denoising effect of the filter depends on the type of noise present in the image. Compared with the existing linear and nonlinear filtering methods, the performance of the proposed improved Wiener filter in most noise models is relatively better. But the Wiener filter needs the spectrum information of the original signal and noise, and it can only achieve good results when the signal is sufficiently smooth [17]. The spatial domain denoising algorithm directly performs corresponding processing on the image pixels. According to the type of filter, it can be divided into linear filters and nonlinear filters. Images generally have such a property: the pixel value at any position in an image is closely related to the pixel value in the neighborhood where the pixel is located, such as spatial correlation or similar pixel values [18].

For the transform domain image denoising algorithm, the image is first transformed into other domains, and then, the coefficients are processed by the properties in the transform domain. Finally, the inverse transform is used to reconstruct the coefficients to obtain the denoised image [19]. There are many ways to transform an image from the spatial domain to the transform domain, such as Fourier transform, cosine transform, and Walsh-Hadamard transform. One of the most commonly used is wavelet transform. The wavelet domain spatial adaptive FIR Wiener filtering method proposed in [20] only performs Wiener filtering in each scale. Although it can quickly remove noise, the processing of different types of noise needs to be strengthened [21].

In addition to traditional spatial and frequency domain image denoising algorithms, literature [22] proposes a dual-domain image denoising (DDID) algorithm, using the idea of combining the space domain and the frequency domain, combined with bilateral filtering and short-time Fourier transform to denoise the image hierarchically. After the algorithm is denoised, the image can retain the original image details to a greater extent and obtain better visual effects. The DDID algorithm divides the noisy image into the base layer and the detail layer to process separately and realizes the image detail enhancement with good effect. Therefore, since the algorithm was proposed, it has been widely used in image denoising. However, the boundary information on the multimode image cannot effectively suppress the negative ringing effect, and the detail preservation needs to be improved [23].

In recent years, deep learning algorithms have been rapidly developed, and the convolution neural network (CNN) method has been proposed to use a layer-by-layer initialization method to overcome difficult problems in the training process. CNN has been widely used in the field of computer vision and has significant effects on solving image classification, target detection, and image recognition problems [24]. With the needs of research, the neural network structure is continuously deepened to build a higher and more accurate deep learning network. Because CNN can directly input the original image, it is simple and easy to use, is widely recognized by the academic community, and has been successfully used in the field of image denoising. Reference [25] comprehensively studies the most advanced image denoising methods using CNN. A denoising prior driven network (PDNN) is proposed to remove fixed-level Gaussian noise. In the BSD-68 and Set-12 datasets, PDNN shows good denoising results in terms of PSNR. In some cases, combining neural networks with traditional methods can achieve better results. For example, literature [26] uses the powerful nonlinear fitting ability of a neural network to combine a neural network with a wavelet method. A neural network is used to find the optimal coefficients of Gabor wavelet, and a neural network can adaptively select wavelet parameters; a combination of RBF network and wavelet is trained. This method has a good effect in the field of sound signal detection, and the theoretical effect of image denoising needs further practical verification.

Because the image is often contaminated by noise and becomes blurred, the image obtained by the above algorithm still has the problem of a blurred image and unsatisfactory effect. Therefore, a multifeature extraction algorithm based on the depth residual network is proposed for medical MR image denoising. The innovation of the proposed method is as follows:

1. In order to improve the learning ability of the image denoising algorithm and reduce the time of model training, multifeature extraction technology is adopted. Three different convolution kernels of different sizes are used to extract features from the input image in a way that the center position is unchanged and synchronized to obtain richer image features and achieve a better denoising effect
2. Due to the large number of layers of the deep neural network, backward propagation easily leads to the disappearance of the gradient, making the training result poor. The proposed algorithm introduces residual learning and learns image noise residuals based on function mapping, thereby achieving image denoising and accelerating and optimizing the deep network. Especially under high-intensity noise levels, the denoising advantage is more prominent

## 3. Denoising Network

### 3.1. Multifeature Extraction Residual Network Denoising Framework

Since image denoising is a typical restoration problem, the proposed denoising network model uses a fully convolutional layer network, which removes the pooling layer in a conventional network. The function of dimensionality reduction and parameter reduction is accomplished by learning residual mapping. The multifeature extraction residual network denoising framework is shown in Figure 1.

The first layer uses multiple feature extraction layers to extract different feature information and map the input image from image space to feature space. After that, a series of residual units are connected in series to form a chain structure, and then the residual image containing only noise information is generated by the last convolution layer reconstruction. Finally, the final denoising result is calculated by the global skip connection. For the loss function in training, the joint loss function which combines the traditional mean square error loss and the perceptual loss is used. The perceptual loss is defined and calculated by a pretrained network [27].

### 3.2. Residual Learning

For the general convolution neural network, image denoising problems are adopted by learning the clean image way. The image result calculated by the network is compared with the standard image, and the cost function is to minimize this error. The formula is as follows:

(1) $$\begin{array}{c} J\left(\theta \right)=\frac{1}{m}\overset{m}{\underset{i}{\sum }}\left(\frac{1}{2}{\left\|h_{w,b}\left(x^{\left(i\right)}\right)-y^{\left(i\right)}\right\|}^{2}\right), \end{array}$$

where *x* stands for the standard image, *y* represents the image after network calculation, and *m* represents the number of images. For the entire network, the cost function obtained by learning noise images is determined by *h*_*w*,*b*_(*x*^(*i*)^) − *y*^(*i*)^.

For the whole model, residual learning is a very important technology. Many network models predict a clean image without pollution by learning mapping functions [28]. For residual learning, it is based on *R*(*y*) ≈ *v* function mapping learning image noise residual and then realizes image denoising. Finally, by using the expected noise residual value and the estimated noise residual value calculated by the convolutional network, the mean square error is obtained, and the cost function of the entire network is obtained. The formula is as follows:

(2) $$\begin{array}{c} L\left(\vartheta \right)=\frac{1}{2n}\overset{n}{\underset{1}{\sum }}{\left\|R\left(y_{i};\vartheta \right)-\left(y_{i}-x_{i}\right)\right\|}_{F}^{2}, \end{array}$$

where *ϑ* represents the training parameter and *n* represents the image block divided into the entire input image. In the network model, this residual learning strategy is selected because it is easier to be optimized by convolutional neural networks and can be very well applied to deep networks. Deep networks face many difficulties, and they are generally very difficult to train. It is mainly reflected in the fact that when the number of layers increases, the backward propagation easily causes the gradient to disappear, making the training result very poor. And this deep residual network solves this problem in the neural network structure, so that the network can be very deep, and the gradient will not disappear. When the noise level is relatively low, the feature map *F*(*y*) = *x* of learning clean images is closer to the initial identity map than the feature map *R*(*y*) ≈ *v* of residual learning. It is equivalent to the mapping relationship of *F*(*y*) = *x* during deep network training, which will make the gradient disappear more easily. Therefore, the residual training will be more conducive to the acceleration and optimization of the deep network.

### 3.3. Batch Normalization

Batch normalization (BN) is an adaptive heavy parameter method, which is mainly used to solve the problem of internal covariate shift (ICS) in deep learning. The model is shown in Figure 2.

The BN model selects *m* inputs because the whole is approximately the same distribution, and *h* obtained as a whole is put into the neural network for batch training. This batch processing method is very beneficial for deep learning, making the model simpler, and solving the problem of difficulty in training after the number of network layers becomes deeper.

For ICS problems that appear in deep network training, the conditional probabilities are consistent, and the marginal probabilities are inconsistent. For all *x* ∈ *X*, the relationship between the conditional probability *P*_*t*_ and the marginal probability *P*_*b*_ is

(3) $$\begin{array}{c} P_{b}\left(Y\left|X=x\right.\right)=P_{t}\left(Y\left|X=x\right.\right),\\ P_{b}\left(X\right)\neq P_{t}\left(X\right). \end{array}$$

Before passing the input vector *x* to the neuron, it should be noted that *x* here not only refers to the input of the input layer but also refers to any input layer or hidden layer in the network. *X* can also be understood as a small batch activation function of a certain layer that needs to be standardized. Translate and scale it first, so that the distribution of *x* becomes a standard distribution normalized in a fixed interval. For the general change framework, it is as follows:

(4) $$\begin{array}{c} h=f\left(g\cdot \frac{x-\gamma }{\kappa }+\upsilon \right), \end{array}$$

where *γ* is the translation parameter, *κ* is the scaling factor, *υ* is the retranslation parameter, and *g* is the rescaling parameter. Through the scaling and translation transformation of *γ* and *κ*, we get the following results:

(5) $$\begin{array}{c} \hat{x}=\frac{x-\gamma }{\kappa }. \end{array}$$

The data obtained satisfy the standard distribution with a mean of 0 and a variance of 1. Substituting formula (5) into formula (4), it is easier to get further transformation:

(6) $$\begin{array}{c} y=g\cdot \hat{x}+\upsilon . \end{array}$$

Finally, a distribution that satisfies the mean *υ* and the variance *g*^2^ is obtained.

This normalization of BN is for a single neuron. When training the network, train a small batch of overall data and then calculate the mean and variance of neuron *x*_*i*_ as

(7) $$\begin{array}{c} \mu_{i}=\frac{1}{m}\sum x_{i},\\ \sigma_{i}=\sqrt{\frac{1}{m}\sum {\left(x_{i}-\mu_{i}\right)}^{2}+\varepsilon }, \end{array}$$

where *m* is the size of the small batch and *ε* is a very small positive value.

### 3.4. Multiple Feature Extraction

In the neural network model, usually in the first layer of connection, multiple identical convolution kernels are generally used to extract shallow features of the image. There are more commonly used convolution kernels such as 1 × 1, 3 × 3, 5 × 5, 7 × 7, and 9 × 9. These convolution kernels are all odd convolution kernels, because this kind of convolution kernel has a common feature. They all have a center point, and even-numbered convolution kernels do not have this property. In shallow feature extraction, usually a larger convolution kernel can learn richer feature information. But the cost is that once the convolution kernel increases, it will adversely affect the training efficiency and speed of the deep network [29].

The proposed algorithm integrates several convolution kernels of different sizes, and its principle is shown in Figure 3. Use multifeature extraction technology to scan the input image block. Since different convolution kernels can extract image features with different information, the one with the largest convolution kernel is used as the moving reference for synchronous movement. In this way, a variety of different feature information will be obtained, and the size of this output is also the same. In the first layer, this feature information is connected in series. Because more feature information is obtained, this multifeature extraction technology greatly improves the training speed in actual model training and greatly improves the convergence speed of the model.

In the first layer of the network, three convolution kernels of different sizes are used, 3 × 3, 5 × 5, and 7 × 7, and the numbers of these three convolution kernels are 12, 20, and 32, respectively. The number has increased sequentially because the 7 × 7 convolution kernel can learn relatively richer features. There are a total of 64 convolution kernels of three different sizes. The three convolution kernels of 3 × 3, 5 × 5, and 7 × 7 are used to scan to the right with a sliding step of 7 in a way that the center position is superimposed. According to this rule, three mapping feature maps with the same size should be obtained [30]. The proposed algorithm passes through the first layer and obtains 64 feature maps of the same size. In the first-level feature extraction, the design of such multiple feature extraction can extract richer image features, which greatly improves the convergence speed and training speed of the network model.

### 3.5. Activation Function

At present, most deep neural networks use a Rectified Linear Unit (ReLU) activation function to accelerate the convergence of the network. The ReLU activation function is not a symmetric function, and the average response of the sequence in ReLU will be less than 0. In addition, even if the input or weight obeys a symmetrical distribution, the response distribution is still asymmetrical. These properties will directly affect the convergence and performance of the network. Therefore, an improved activation function Parametric Rectifier Linear Unit (PReLU) is used. PReLU function is defined as follows:

(8) $$\begin{array}{c} f\left(y_{i}\right)=\left\{\begin{array}{c} y_{i},y_{1}>0,\\ k_{i}y_{i},y_{i}\leq 0, \end{array}\right. \end{array}$$

where *y*_*i*_ is the input of the nonlinear activation function *f* on the *i*th channel and *k*_*i*_ controls the slope of the negative part. When *k*_*i*_ is equal to 0, it becomes the ReLU activation function.

### 3.6. Joint Loss

The pixel-by-pixel loss is usually used as loss function, and the difference between the pixels between the output image and the input image is calculated as the minimization target to obtain a higher signal-to-noise ratio index. However, the output image using the method of comparing the difference pixel by pixel is prone to problems such as excessive smooth and blurry edges. In response to this problem, there are currently many studies showing that comparing the perceived loss of semantic feature level with the image quality perceived by the human eye shows a good uniformity. More edge texture details in real images can be reconstructed, thereby improving some of the problems of the pixel-by-pixel method. However, simply using this loss may also cause problems such as slight color artifacts due to uneven pixel space coverage. Therefore, by combining the two losses to obtain better results, the joint loss *L*_&_ is proposed as

(9) $$\begin{array}{c} L_{\&}=L_{\text{MSE}}+\lambda L_{\text{VGG}}, \end{array}$$

where *L*_MSE_ and *L*_VGG_, respectively, represent the mean square error (MSE) function of pixel-by-pixel comparison and the perceptual loss of feature comparison.

#### 3.6.1. MSE Loss Function

The pixel-by-pixel loss function uses the traditional MSE method to calculate the MSE of the real target and the predicted target. By comparing each pixel to learn the difference between the two, the optimal solution is obtained. The formula is as follows:

(10) $$\begin{array}{c} L_{\text{MSE}}=\frac{1}{N}\overset{N}{\underset{n=1}{\sum }}{\left\|F\left(x\right)-\left(x-y\right)\right\|}_{2}^{2}, \end{array}$$

where *N* is the total number of training samples, *x* is the noise input, *y* is a clean real label, and *F* is the optimal mapping function obtained after training.

#### 3.6.2. Perceptual Loss Function

The realization of the perceptual loss needs to effectively extract the rich and abstract semantic feature information in the image. A pretrained classification network Visual Geometry Group (VGG) is connected in series as a loss network to extract the required feature map definition *L*_VGG_. After the loss network is determined, the loss comparison learning method can input the output *x* − *F*(*x*) and the real noise-free label image *y* through the initial processing of the front-end multifeature extraction residual network into the VGG network. Extract the feature images of the two from one of the convolutional layers *φ* and calculate the Euclidean distance between the semantic features of the two according to the formula. The formula is as follows:

(11) $$\begin{array}{c} L_{\text{VGG}}=\frac{1}{N}\overset{N}{\underset{n=1}{\sum }}{\left\|\varphi_{i}\left(x-F\left(x\right)\right)-\varphi_{i}\left(y\right)\right\|}_{2}^{2}, \end{array}$$

where *φ* is the PReLU function after the *i*th convolutional layer in the loss network. It is used to extract feature maps, using rich edge texture features and semantic information for comparison. The application of joint perception loss in the algorithm is shown in Figure 4.

For joint perception loss, first input the noise image to be processed into the built VGG and train the network through MSE loss. Compare the difference between the learning prediction result and the true label map from the pixel level. At this time, the image output by the network has completely removed the noise points, but the edge information is fuzzy [31]. So, the fuzzy denoising result and label are passed through the pretrained VGG again. The feature maps of the two are obtained from the activation function after the specific convolutional layer for comparison. Minimize the perceptual loss as the training goal for network training, so that the output image contains more edge information features. It is possible to restore the originally blurred area during reconstruction, obtain clearer and sharper image edges, and obtain clearer image denoising results.

## 4. Network Parameter Setting

In the process of neural network training, it is necessary to learn a set of optimal parameters to minimize the result of loss function, so a suitable optimization algorithm needs to be added. So far, the commonly used neural network optimization algorithm is the gradient descent algorithm, which is used to find the minimum parameter of the loss function. In the training process, the error is gradually reduced and the local minimum of the function is found. Differentiate the loss function to get the gradient of a given point [32]. The positive and negative values of the gradient indicate an increase or decrease in the value of the loss function. Select the direction that reduces the cost function value, that is, the negative gradient direction, multiply the updated amount of the parameter calculated by the learning rate, and update the parameter.

The single-step weights and biases are updated as follows:

(12) $$\begin{array}{c} \omega_{k}\to \omega_{k}=\omega_{k}-\partial \frac{\delta C}{{\delta \omega }_{k}},\\ b_{l}\to b_{l}=b_{l}-\partial \frac{\delta C}{\delta b_{l}}. \end{array}$$

The main problem of the gradient descent algorithm is that if the location of the initial point is unreasonably selected, the network is easy to fall into a local optimum, and it is difficult to find the global optimum. In addition, if the step size of the single step down is too small, the calculation amount will be too large, and if the number of iterations is too large, the step size may be too large to skip the optimal solution. And the gradient descent algorithm is not fast enough when the amount of data is large. Therefore, the stochastic gradient descent (SGD) algorithm is used to calculate the gradient using a single sample to speed up the calculation. However, the SGD method uses individuals to represent the overall change trend and cannot ensure that each iteration tends to the global optimal solution, and it cannot guarantee that each iteration will reduce the loss function result. Therefore, an adaptive moment estimation (Adam) optimization algorithm is proposed to replace the SGD algorithm [33]. The SGD algorithm maintains a single learning rate, updates all weights, and keeps the learning rate during the training process unchanged. And Adam iteratively updates the neural network weights by calculating the first-order moment estimation and the second-order moment estimation of the gradient. The adaptive learning rate is calculated for each parameter to solve the problem of high-intensity noise or sparse gradient [34]. The basic steps of the Adam optimization algorithm are as follows:

**Step 1 .**

Suppose *f*(*θ*) is the noise objective function, which is a random scalar function with differentiable parameters *θ*.

**Step 2 .**

Update the exponential moving average *s*_*t*_ and squared gradient *v*_*t*_ of the gradient. The moving average is estimated using the first-order moment and the second-order original moment of the gradient, and the step size *ζ* is selected reasonably.

**Step 3 .**

Initialize the deviation correction term to obtain the gradient of the random objective function *f*. Then, use the exponential moving average of *v*_*t*_ and the decay rate *τ*_2_ to estimate the second-order original moment. That is, eliminate *v*_*t*_:

(13) $$\begin{array}{c} v_{t}=\left(1-\tau_{2}\right)\overset{t}{\underset{i=1}{\sum }}\tau_{2}^{t-i}\cdot q_{i}^{2}, \end{array}$$

where *τ*_2_ is the exponential decay rate estimated by the second moment, *t* is the time step, and *q*_1_, ⋯, *q*_*T*_ is the gradient on the time step sequence. In order to understand how the expected value penalty *E*[*v*_*t*_] of the exponential moving average at time step *t* is related to the true second moment, the deviation between these two quantities is corrected, as follows:

(14) $$\begin{array}{c} E\left[v_{t}\right]=E\left[\left(1-\tau_{2}\right)\overset{t}{\underset{i=1}{\sum }}\tau_{2}^{t-i}\cdot q_{i}^{2}\right]=E\left[q_{t}^{2}\right]\cdot \left(1-\tau_{2}\right)\overset{t}{\underset{i=1}{\sum }}\tau_{2}^{t-i}+\varepsilon =E\left[q_{t}^{2}\right]\cdot \left(1-\tau_{2}^{t}\right)+\varepsilon . \end{array}$$

If the second moment *E*[*q*_*t*_^2^] is static, then *ε* = 0.

In addition, for the parameter settings during training, the input of the network is to randomly cut out 45 × 45 image blocks from the training set images. The first layer of the network consists of convolution kernels of multiple sizes. Among them, there are 12 convolution kernels of 3 × 3, 20 convolution kernels of 5 × 5, 32 convolution kernels of 7 × 7, and a total of 64 channels. For the convolutional layer in the following residual module, 64 convolution kernels of 3 × 3 are uniformly used. The last reconstruction layer uses *c* convolution kernels of 3 × 3 (*c* = 1 for grayscale images, *c* = 3 for color images). The algorithm to optimize the regression target uses the Adam method, and the momentum parameter is 0.9. When the training function is joint loss, the training batch size is smaller than 18, and the initial learning rate is 10-4. The learning rate is halved after every 2.0 × 105 iterations.

In the batch normalization used, a sufficient comparison experiment was done on the settings of the minibatch parameters. In the comparative experiment, the minibatch size is set to 32, 64, and 128, respectively, and the model convergence speed and the final denoising effect achieved under these parameters are compared. It is found from the experimental results that the overall effect of image denoising is the best when the minibatch value is 64. Therefore, in the training process of the denoising model, the value of batch-normalized minibatch is set to 64.

## 5. Experiment Scheme and Result Discussion

In order to evaluate the proposed algorithm, we must first have an evaluation standard and do different experiments on different test datasets, fully contrast with other excellent image denoising algorithms, and finally draw a conclusion.

### 5.1. Experimental Dataset

Since the use of the deep residual network algorithm requires a large amount of training image data, the experimental data selected by the proposed algorithm uses the internationally published glioblastoma multiforme (GBM) multimodal MR image dataset TCGA. Among them, the foreign population GBM experimental test library (TCGA-GBM) and the Chinese population GBM experimental test library (CH-GBM) are established. Some image examples of the dataset are shown in Figure 5.

In the experiment, 227 images were randomly selected from the TCGA-GBM dataset, of which 200 were used as training images and the remaining 27 were used as test images. The image size is set to 180 × 215 and 64 × 77. 115 images were randomly selected from the CH-GBM dataset, 100 were used as training images, and the remaining 15 were used as test images. The image size is set to 180 × 215 and 64 × 77. The image block size is set to 32 × 32, and the image block step size is 10. A total of about 86,000 training image blocks can be obtained. Then, the tested images are evaluated using the Peak Signal Noise Ratio (PSNR) and Structural Similarity Index (SSIM).

In the proposed algorithm, the size of the training set is artificially increased by methods such as image translation and flipping. Because in the training process, when the amount of data is small, it will cause the model to overfit, so that the training error is small and the test error is large. Therefore, the occurrence of overfitting can be effectively suppressed by adding a regular term after the cost function.

### 5.2. Evaluation Standard of Denoising Effect

The proposed algorithm mainly uses two objective evaluation indexes: PSNR and SSIM. Given a reference image, it is represented by *f*, and the test image is represented by *d*. The size of these two images is (*M* × *N*); then, the PSNR between the images is defined as

(15) $$\begin{array}{c} \text{PSNR}\left(f,d\right)=10\log_{10}\frac{255^{2}}{\text{MSE}\left(f,d\right)},\\ \text{MSE}\left(f,d\right)=\frac{1}{MN}\overset{M}{\underset{i=1}{\sum }}\overset{N}{\underset{j=1}{\sum }}{\left(f_{ij}-d_{ij}\right)}^{2}. \end{array}$$

When MSE tends to zero, the value of PSNR tends to infinity. This means that the higher the PSNR value, the better the image quality. The smaller the PSNR value, the greater the difference between the two images.

SSIM is a quality evaluation model that takes into account the brightness distortion, contrast distortion, and related loss of the image. It is defined as

(16) $$\begin{array}{c} \text{SSIM}\left(f,d,l\right)=l\left(f,d\right)c\left(f,d\right)s\left(f,d\right),\\ \left\{\begin{array}{c} l\left(f,d\right)=\frac{2\mu_{f}\mu_{d}+C_{1}}{\mu_{f}^{2}+\mu_{d}^{2}+C_{1}},\\ c\left(f,d\right)=\frac{2\sigma_{f}\sigma_{d}+C_{2}}{\sigma_{f}^{2}+\sigma_{d}^{2}+C_{2}},\\ s\left(f,d\right)=\frac{\sigma_{fd}+C_{3}}{\sigma_{f}\sigma_{d}+C_{3}}, \end{array}\right. \end{array}$$

where *l*(*f*, *d*) is the brightness comparison function, used to calculate the similarity of the average brightness *μ*_*f*_ and *μ*_*d*_ of the two images. When *μ*_*f*_ = *μ*_*d*_, *l*(*f*, *d*) takes the maximum value. *c*(*f*, *d*) is the contrast comparison function. Measure the similarity of the contrast of two images. Contrast is measured by standard deviation *σ*_*f*_ and *σ*_*d*_. It is only when *σ*_*f*_ equals *σ*_*d*_ that *c*(*f*, *d*) has a maximum value of 1. *s*(*f*, *d*) is a structure comparison function, used to represent the correlation between *f* and *d* pixels of two images. *σ*_*fd*_ is the covariance between *f* and *d*, and the value range of SSIM is [0,1]. A value of 0 means that there is no correlation between the two images, and a value of 1 means that *f* is equal to *d*. Constants *C*_1_, *C*_2_, and *C*_3_ are used to avoid the phenomenon of a zero denominator.

### 5.3. Analysis of Network Iteration Algorithm

For the proposed network, the training iterations are all 50. When image denoising, the learning rate that is too small will lead to slower convergence speed, and the long-term slowness in feature learning will cause weak noise in the parameter update process, which will affect the quality of the denoised image. However, when the learning rate is large, the network system will be unstable. Considering comprehensively, the learning rate of the proposed network model is 0.01. The MatConvNet toolkit is used to train the model in the network. Since the training time of each model is different, the proposed training model runs for two days on average when different noises are added.

In order to effectively obtain the spatial information of the image, a 15-layer network is set up, including the convolutional layer, activation function, pooling layer, and BN layer. Under the condition that the basic parameters of the experiment remain unchanged, the influence of the two optimization algorithms of Adam and SGD on the denoising results is studied. When the image is added with 7% noise, the average PSNR value of the test image after denoising using the model optimized by Adam and SGD algorithm is shown in Figure 6.

It can be seen from Figure 6 that the proposed network model using the Adam algorithm optimized model to remove the noise in the medical MR image is better than the SGD algorithm optimized model. The average PSNR value has increased by about 1 dB, and the denoising result is relatively stable. When the number of iterations is 20, the average PSNR value tends to be stable. Therefore, in the proposed network model, the optimization algorithm uses Adam.

### 5.4. Qualitative Comparison of Denoising Effects

In order to compare the effect of medical MR image size on the denoising effect, the same TCGA-GBM dataset images with sizes of 190 × 215 and 62 × 77 were selected in the experiment. Train the denoising algorithm by manually adding 7% of noisy images. Finally, four different MR images are selected as test images to obtain the final denoising image.  Figure 7 shows the average PSNR curve after denoising the two different sizes of test images.

It can be seen from Figure 7 that image training models of different pixels have a relatively large impact on the denoising effect. When training the model with images with larger pixels, the PSNR of the denoised image is significantly higher than that of images with smaller pixels. When the pixels are small, the average PSNR of the training model after denoising the image is relatively low, the whole process is unstable, and the convergence speed is slow. When the pixels are small, this is equivalent to reducing the amount of training image data. This leads to overfitting of the model, which makes the training error smaller and the test error larger. Therefore, when training the model, choosing a larger amount of data will help improve denoising performance of the algorithm. Through analyzing the influence of the above-mentioned selected network parameters on the image denoising performance, in the verification experiment of the proposed algorithm, both the training image and the test image are selected in the size of 190 × 215, and the optimization algorithm is Adam.

In order to further visually demonstrate the denoising effect of the proposed algorithm on the TCGA-GBM and CH-GBM datasets, compare it with literature [14, 20, 26]. The result is shown in Figure 8.

It can be seen from Figure 8 that, compared with the other three denoising algorithms, the image after denoising by the proposed algorithm is more thorough and the edge preservation effect is better. In contrast, the image denoised by the algorithm in literature [14, 20] obviously has some residual noise, and the noise removal is not very thorough. In the literature [14], the image edge blur after denoising using the improved MMF algorithm is larger. In particular, the blurred residual noise can be clearly seen around the edge of the brain image. And for the smoother part of the original image, the image becomes unsmooth after denoising, and fuzzy noise blocks of varying degrees appear. However, in the literature [20], the adaptive FIR algorithm is used to denoise the denoised image twice, and the phenomenon of filtering will appear. But for the Rician noise in medical MR images, the denoising image produces blurring, which makes the image noise removal incomplete. The main manifestation is that there are noise points around the edges of the image, but it is improved compared to the improved MMF algorithm. In Reference [26], combining the neural network and wavelet method, the image after denoising is significantly improved compared with the previous two methods. However, this method smoothes the details of the image, especially the contour area of the brain image, and the phenomenon of excessive filtering occurs, thereby losing useful information in the details. The proposed algorithm has a relatively good effect on removing noise in medical MR images, avoids the problem of incomplete denoising of the first two denoising methods, and can also reduce oversmoothing. Compared with the three comparison algorithms, it has a better overall effect on noise removal.

### 5.5. Quantitative Comparison of Denoising Effects

Aiming at the problem of denoising in medical MR images, the denoising effects of different denoising algorithms are clearly analyzed. The proposed algorithm and the algorithm in literature [14, 20, 26] are quantitatively evaluated in two indicators: average PSNR and SSIM. Among them, the average SSIM of the four denoising algorithms after denoising the medical MR image with different noise intensities is shown in Table 1.

It can be seen from Table 1 that the SSIM value of the proposed algorithm is significantly higher than that of the algorithm in [14, 20], and the denoising effect is consistent with the subjective observation results. Comparing the proposed algorithm with the algorithm in [26], both have improved. Especially when the noise intensity is relatively weak, the SSIM value of the proposed algorithm has been greatly improved, showing a very obvious advantage. Therefore, the proportion of useful information in the denoised image of the proposed algorithm is closer to that of the original noise-free image. When 1% noise is added, SSIM can reach 0.9941 after denoising. Compared with other algorithms, the values are improved, and more satisfactory results are obtained, with less information loss.

On the TCGA-GBM and CH-GBM datasets, for different noise levels, the proposed algorithm is quantitatively compared with the MR image denoising effect of the algorithms in [14, 20, 26]. The average PSNR and SSIM curves obtained are shown in Figures 9 and 10.

It can be seen from Figures 9(a) and 10(a) that under different noise intensities, the average PSNR of the image after denoising using the proposed algorithm is significantly higher than that of the image processed by other denoising algorithms. And when denoising weakly noisy images, the average PSNR of the proposed algorithm and other contrasting algorithms are relatively small. In the case of strong noise denoising, the average PSNR is quite different, indicating that the proposed algorithm has better effect on removing strong noise in MR images. The denoised image has a very high similarity to the original noiseless image.

At the same time, it can be seen from Figures 9(b) and 10(b) that the four denoising algorithms have little difference in the average SSIM of the image after denoising when the noise intensity is weak. When the noise intensity is high, the average SSIM of the proposed algorithm after denoising shows obvious advantages. In terms of structural similarity, it is closer to the original image.

In summary, the proposed algorithm is better than the other three denoising algorithms in denoising simulated medical MR images. Especially under strong noise, it can effectively remove the noise in the simulated medical MR image.

## 6. Conclusions

Currently, medical image information can be obtained through a variety of technical means, among which MRI is a relatively common medical image acquisition technology. However, MR images will be interfered by random noise during the acquisition process, which reduces the useful information in images. Decreasing the accuracy and effectiveness of imaging will directly affect the correct diagnosis and treatment of clinicians. Therefore, a denoising algorithm for medical MR images based on multifeature extraction based on a deep residual network is proposed. The feature extraction layer is constructed by combining three convolution kernels of different sizes to obtain multiple shallow features for fusion and combined with batch normalization and residual learning technology to accelerate and optimize the deep network. In addition, a joint loss function is defined by combining the perceptual loss and the traditional mean square error loss to generate a clearer target image. Based on the MATLAB simulation platform, the TCGA-GBM and CH-GBM datasets are used to experimentally demonstrate the proposed algorithm. The results show that the performance of the proposed algorithm is the best when the image size is set to 190 × 215 and Adam is selected as the optimization algorithm. And the two indexes of PSNR and SSIM of the proposed algorithm are significantly higher than other comparison algorithms. As the noise level increases, the difference between the values becomes larger, which shows that it is suitable for processing high-intensity noise MR images.

Regardless of whether it is in the classification or denoising of deep residual learning, the parameter adjustment of the deep network has always been a key step, and it is more difficult. Therefore, further research is needed. In addition, the deep residual network can achieve better results when the amount of training data is large. But when the amount of data is small, the denoising effect needs to be improved. At the same time, the amount of data is large, which is slower than traditional algorithms. Therefore, the training speed of the network needs to be further improved while ensuring the denoising effect.

## Figures and Tables

**Figure 1:** Multifeature extraction residual network denoising framework.

**Figure 2:** The structure of BN model.

**Figure 3:** Structure of multifeature extraction model.

**Figure 4:** Flow chart of joint loss.

**Figure 5:** Partial image examples of the dataset.

**Figure 6:** Denoising results using different optimization algorithms.

**Figure 7:** Denoising results of different size images.

**Figure 8:** Comparison of denoising effects of different algorithms.

**Figure 9:** Comparison of denoising effects of different algorithms in the TCGA-GBM dataset.

**Figure 10:** Comparison of denoising effects of different algorithms in the CH-GBM dataset.

**Table 1:** SSIM comparison of different denoising algorithms.

Dataset	Algorithm	1%	4%	7%	10%	13%
TCGA-GBM	Ref. [14]	0.9903	0.9584	0.9153	0.8612	0.8109
	Ref. [20]	0.9901	0.9592	0.9276	0.8928	0.8529
	Ref. [26]	0.9918	0.9643	0.9374	0.9022	0.8657
	The proposed algorithm	0.9941	0.9668	0.9417	0.9152	0.8893

CH-GBM	Ref. [14]	0.9829	0.9622	0.9238	0.8874	0.8378
	Ref. [20]	0.9923	0.9637	0.9246	0.8984	0.8557
	Ref. [26]	0.9935	0.9626	0.9415	0.9043	0.8736
	The proposed algorithm	0.9978	0.9689	0.9426	0.9037	0.8809

## Data Availability

The data included in this paper are available without any restrictions.
